The article "Hydroxychloroquine in the Treatment of COVID-19: A Multicenter Randomized Controlled Study" was retracted in 2022. Reasons: duplicated data; unreliable data; concerns about the data.

# Hydroxychloroquine in the Treatment of COVID-19: A Multicenter Randomized Controlled Study

**DOI:** 10.4269/ajtmh.20-0873

**Published:** 2020-08-14

**Authors:** Sherief Abd-Elsalam, Eslam Saber Esmail, Mai Khalaf, Ehab Fawzy Abdo, Mohammed A. Medhat, Mohamed Samir Abd El Ghafar, Ossama Ashraf Ahmed, Shaimaa Soliman, Ghada N. Serangawy, Mohamed Alboraie

**Affiliations:** 1 Department of Tropical Medicine and Infectious Diseases, Faculty of Medicine, Tanta University, Tanta, Egypt;; 2 Department of Gastroenterology and Tropical Medicine, Faculty of Medicine, Assiut University, Assiut, Egypt;; 3 Department of Anesthesia, Surgical Intensive Care and Pain Medicine, Faculty of Medicine, Tanta University, Tanta, Egypt;; 4 Department of Internal Medicine, Ain-Shams University, Cairo, Egypt;; 5 Public Health and Community Medicine, Menoufia University, Menoufia, Egypt;; 6 Department of Forensic Medicine and Toxicology, Faculty of Medicine, Tanta University, Tanta, Egypt;; 7 Department of Internal Medicine, Al-Azhar University, Cairo, Egypt

## Abstract

The COVID-19 pandemic is showing an exponential growth, mandating an urgent need to develop an effective treatment. Indeed, to date, a well-established therapy is still lacking. We aimed to evaluate the safety and efficacy of hydroxychloroquine (HCQ) added to standard care in patients with COVID-19. This was a multicenter, randomized controlled trial conducted at three major university hospitals in Egypt. One hundred ninety-four patients with confirmed diagnosis of COVID-19 were included in the study after signing informed consent. They were equally randomized into two arms: 97 patients administrated HCQ plus standard care (HCQ group) and 97 patients administered only standard care as a control arm (control group). The primary endpoints were recovery within 28 days, need for mechanical ventilation, or death. The two groups were matched for age and gender. There was no significant difference between them regarding any of the baseline characteristics or laboratory parameters. Four patients (4.1%) in the HCQ group and 5 (5.2%) patients in the control group needed mechanical ventilation (*P* = 0.75). The overall mortality did not differ between the two groups, as six patients (6.2%) died in the HCQ group and 5 (5.2%) died in the control group (*P* = 0.77). Univariate logistic regression analysis showed that HCQ treatment was not significantly associated with decreased mortality in COVID-19 patients. So, adding HCQ to standard care did not add significant benefit, did not decrease the need for ventilation, and did not reduce mortality rates in COVID-19 patients.

## INTRODUCTION

Coronaviruses are a large family, which may cause illness in animals or humans. In humans, several coronaviruses are known to cause respiratory infections, ranging from common cold to more severe diseases such as Middle East respiratory syndrome and SARS.^1–6^ The most recently discovered coronavirus is SARS-CoV-2 which causes COVID-19. As cases of COVID-19 continue to rise in different countries, health systems are facing enormous pressure to manage COVID-19 patients. By August 2, 2020, COVID-19 has been confirmed in about 17,660,523 million individuals worldwide and has resulted in more than 680,894 deaths. These numbers are still increasing. More than 180 countries have reported laboratory-confirmed cases of COVID-19 on all continents, except Antarctica.^1–4^ In Egypt, the official number of infected patients was 94,316, with 4,834 deaths as of August 2, 2020.^1–11^

Although many vaccines are in development, effective therapy is needed to treat currently infected patients and prevent mortality. Chloroquine (CQ) and hydroxychloroquine (HCQ) have been used for decades in the treatment and prophylaxis of a number of conditions including malaria. The ability of these drugs to inhibit other coronaviruses, such as SARS-CoV-1, has been explored. Although generally considered safe, there are potential risks associated with taking these medications, including cardiac arrhythmia.^7–11^

Although an initial study in France found encouraging results for the treatment of COVID-19 with HCQ, the study was later criticized for its methodological problems, leading to skepticism about the validity of its results. Other similar results were not represented in any further subsequent studies, but even reported deleterious clinical outcomes especially cardiac adverse events like prolongation of QT interval.^8^ On March 28, 2020, the Food and Drug Administration (FDA) granted an emergency use authorization for use of oral formulations of CQ and HCQ in the treatment of COVID-19.^7–11^ Based on emerging data showing CQ and HCQ as unlikely to be effective in the treatment of COVID-19,^12,13^ the FDA revoked its previous emergency use authorization for both drugs on June 15, 2020.

In this study, we aimed to evaluate the safety and efficacy of HCQ added to the standard of care versus the standard of care alone in patients with COVID-19.

## METHODS

Patients admitted to three tertiary referral centers (*n* = 194) managing patients with suspected and confirmed COVID-19 in Egypt in the period between March and June 2020 were enrolled. The patients were clinically stratified into mild, moderate, and severe disease according to the WHO interim guidelines published on March 13, 2020. Mild cases represented patients with uncomplicated upper respiratory tract viral infection, moderate cases represented patients with pneumonia but without need for supplemental oxygen, whereas severe disease represented cases with fever or suspected respiratory infection, plus one of the following: respiratory rate > 30 breaths/min, severe respiratory distress, or SpO_2_ ≤ 93% on room air.^14^

The Egyptian Ministry of Health (MOH) adopted a standard of care treatment protocol for COVID-19 patients. It included paracetamol, oxygen, fluids (according to assessment), empiric antibiotic (cephalosporins), oseltamivir if needed (75 mg/12 hours for 5 days), and invasive mechanical ventilation with hydrocortisone for severe cases if PaO_2_ < 60 mmHg, O_2_ saturation < 90% despite oxygen or noninvasive ventilation, progressive hypercapnia, respiratory acidosis (pH < 7.3), and progressive or refractory septic shock.^15^

Patients were randomized into two groups using a computerized random number generator using simple randomization with an equal allocation ratio. During randomization, the proportional allocation of each clinical stratum was equalized in both groups.

### Study groups.

1. Hydroxychloroquine group: This group included 97 patients who received HCQ 400 mg twice daily (in day 1) followed by 200 mg tablets twice daily added to the standard of care treatment adopted by the Egyptian MOH for 15 days.
2. Control group: This group included 97 patients who received only the standard of care treatment adopted by the national MOH for 15 days.

All the patients were followed up for 4 weeks.

The study included all patients admitted with SARS-CoV-2 infection and enrolled both genders. Patient who had allergy or contraindication to HCQ, pregnant and lactating females, and patients with cardiac problem (chronic heart failure or prolonged QT interval on electrocardiogram [ECG]) were excluded from the study.

Informed written consent was obtained from each participant, and the study was approved by the Ethics Committee of the Faculty of Medicine, Tanta University. Privacy of the participants and confidentiality of the data were assured. Risks and benefits were explained to the patients. The study was registered on clinicaltrials.gov with registration number NCT04353336.

All the participants were subjected to thorough history taking and full clinical examination including age, gender, weight and height measurements, and calculation of body mass index (BMI); medication history; and investigations in the form of complete blood picture, liver function tests, computed tomography of the chest (CT chest), and SARS-CoV-2 detection in nasopharyngeal swabs using PCR and ECG. Assessment of the studied medication side effects was performed using a questionnaire.

### Statistical analysis.

Data were analyzed using Statistical Package for Social Sciences V. 23 and were expressed in number, percentage (%), mean (*x̅*) and SD. The variables were tested for normality by the Shapiro–Wilks test. Student’s *t*-test was used for normally distributed quantitative variables and Mann Whitney’s test for not normally distributed ones. Chi-square test (χ^2^) was used to study association between qualitative variables, and whenever any of the expected cells were less than five, Fischer’s exact test was used. Binary logistic regression was used to ascertain the effect of the potential risk factors on the patients’ mortality. A two-sided *P*-value of < 0.05 was considered statistically significant.

### Post hoc power analysis.

Considering the percentage of recovery as a primary endpoint and by using G*power program, post Hoc power analysis revealed a sample power of 80.6% with the following input parameters: two-tailed α error 0.05, 54.0% recovery rate in the HCQ group, 34.0% recovery in the control group, and 97 sample size in each group.^16^

## RESULTS

At the time of presentation, interrupted fever was present in 44.6%, continuous fever in 22.3%, headache in 42.9%, sore throat in 25.7%, anorexia in 33.1%, anosmia in 26.9%, pallor in 3.4%, cyanosis in 4.6%, fatigue in 49.0%, vomiting in 13.7%, diarrhea in 35.0%, abdominal pain in 19.4%, cough in 61.3%, and dyspnea in 24.2% of the included patients. Oxygen saturation between 95 and 90 was present in 16.0%, 90–85 in 7.4%, and less than 85 in 6.9% of all the participants.

The computed tomography chest scans were normal in 33.1%, ground-glass opacities in 23.4%, confluent opacities in 25.7%, consolidation in 10.9%, extensive consolidation in 6.3%, and emphysema in only 0.6%.

The two groups were matched for age and gender, with no significant difference between them. They had no significant difference regarding BMI, residence, smoking, pregnant females, or the presence of comorbidities. The patients were randomized equally between the two groups regarding the disease severity (Table 1).

**Table 1:** Patients’ characteristics between the two groups

Character	Group 1 (*n* = 97)	Group 2 (*n* = 97)	Total (*n* = 175)	*P*-value
Age (years), mean ± SD	40.35 ± 18.65	41.09 ± 20.07	40.72 ± 19.32	0.80
Range	2.0–85.0	2.0–83.0	–	–
Gender, *n* (%)				
Male	56 (57.7)	58 (59.8)	114 (58.8)	0.77
Female	41 (42.3)	39 (40.2)	80 (41.2)	
Body mass index, *n* (%)				
Normal	4 (4.1)	9 (9.3)	13 (6.7)	0.46
Overweight	32 (33.0)	29 (29.9)	61 (31.4)	
Obese	40 (41.2)	35 (36.1)	75 (38.7)	
Morbid obesity	21 (21.6)	24 (24.7)	45 (23.2)	
Residence, *n* (%)				
Rural	54 (55.7)	46 (37.4)	100 (51.5)	0.25
Urban	43 (44.3)	51 (52.6)	94 (48.5)	
Smoking, *n* (%)	35 (36.1)	25 (25.8)	60 (31.4)	0.12
Comorbidities, *n* (%)	15 (15.5)	12 (12.4)	27 (14.3)	0.53
Liver diseases, *n* (%)	0 (0.0)	2 (2.1)	2 (1.0)	0.50
Renal impairment, *n* (%)	2 (2.1)	4 (4.1)	6 (3.1)	0.68

There was no significant difference between the two groups regarding laboratory parameters (Table 2).

**Table 2:** Laboratory parameters between the two groups

Investigation	Group 1 (*n* = 97), mean ± SD	Group 2 (*n* = 97), mean ± SD	*P*-value
Hemoglobin	13.20 ± 2.00	12.83 ± 1.88	0.19
Platelets	280.78 ± 102.12	252.08 ± 97.03	0.05
White blood cells	5.48 ± 2.82	6.07 ± 3.376	0.82
Lymphocytes	30.14 ± 21.45	31.95 ± 17.00	0.07
Direct bilirubin	0.26 ± 0.11	0.33 ± 0.26	0.09
Indirect bilirubin	0.55 ± 0.20	0.58 ± 0.26	0.46
Albumin	4.06 ± 0.38	3.95 ± 0.45	0.07
Alanine aminotransferase	33.07 ± 23.15	28.17 ± 18.31	0.10
Aspartate aminotransferase	29.52 ± 13.45	26.89 ± 179.25	0.06
International normalized ratio	1.08 ± 0.14	1.06 ± 0.15	0.19
D-dimer	26.74 ± 145.03	28.17 ± 220.11	0.42
Median	0.34	0.32	
Lactate dehydrogenase	291.52 ± 149.47	282.04 ± 179.25	0.07
Median	250.0	230.0	
Ferritin	374.75 ± 469.49	305.14 ± 357.24	0.07
Median	234.0	194.0	
Creatinine	0.94 ± 0.29	0.98 ± 0.27	0.05
C-reactive protein	27.88 ± 48.91	35.86 ± 63.60	0.38
Median	12.0	12.0	

Mechanical ventilation was needed in four patients (4.1%) in the HCQ group and 5 (5.2%) in the control group, with no significant difference between the two groups (*P* = 0.75). Six patients (6.2%) died in the HCQ group, and five patients (5.2%) died in the control group without any significant difference between the two groups either (*P* = 0.76).

Eleven patients (11.3%) in the HCQ group needed intensive care unit (ICU) admission, and 13 patients (13.4%) in the control group needed the same (*P* = 0.83). The mean duration to negative PCR was 17 ± 3 days in the HCQ group and 18 ± 2 in the control group (*P* = 0.11). The HCQ group had a mean of 9 ± 2 days to show clinical improvement and 11 ± 3 days to hospital discharge, whereas the control group had a mean of 10 ± 3 to clinical improvement and 11 ± 2 to hospital discharge (*P* = 0.80 and 0.52, respectively) (Table 3).

**Table 3:** Clinical course in both groups

Clinical course	Hydroxychloroquine (*n* = 97)	Control (*n* = 97)	*P*-value
Disease severity after 28 days, *n* (%)			
Recovered	52 (53.6)	33 (34.0)	0.06
Mild	23 (23.7)	39 (40.2)	
Moderate	8 (8.2)	11 (11.3)	
Severe	8 (8.2)	9 (9.2)	
Death	6 (6.1)	5 (5.1)	
Need for ICU	11 (11.3)	13 (13.4)	0.83
Duration to negative PCR, mean ± SD	17.01 ± 2.98	17.64 ± 2.45	0.11
Duration to clinical improvement, mean ± SD	9.43 ± 1.87	9.52 ± 2.94	0.80
Duration to hospital discharge, mean ± SD	11.04 ± 2.71	11.27 ± 2.19	0.52

After 28 days, there was no significant difference between the two groups regarding the clinical outcome (*P* = 0.07). Complete recovery was achieved in 52 cases (53.6%) of the HCQ group, whereas 23 cases (23.7%) were in mild, 8 (8.2%) were in moderate, 8 (8.2%) in severe disease status, and six patients (6.1%) died. Among the control group, 33 patients (34.0%) recovered completely, 39 (40.2%) were in mild, 10 (10.3%) were in moderate, 9 (9.2%) were in severe disease status, and five patients (5.1%) died.

By logistic regression, the overall mortality was not significantly associated with HCQ therapy; however, it was significantly related to the patient’s age, alanine aminotransferase, serum creatinine, serum ferritin, C-reactive protein, oxygen saturation, and the presence of diabetes mellitus (Table 4).

**Table 4:** Univariate regression of the potential risk factor of mortality

Variable	Univariate			
	*P*-value	OR	95% CI	
			Lower	Upper
Age	< 0.001	1.081	1.035	1.129
Gender	0.736	1.243	0.351	4.396
Smoking	0.997	–	–	–
Alanine aminotransferase	< 0.001	1.047	1.024	1.071
Albumin	0.025	0.201	0.050	0.816
Creatinine	< 0.001	47.506	7.347	307.17
Ferritin	0.002	1.002	1.001	1.003
C-reactive protein	< 0.001	1.029	1.017	1.040
O_2_ saturation	< 0.001			
95–90	0.035	13.739	1.198	157.62
85–90	< 0.001	632.00	51.705	7,725.0
DM	0.001	9.293	2.556	33.792
Hydroxychloroquine treatment	0.757	0.824	0.243	2.797

OR = odds ratio; DM = diabetes mellitus.

## DISCUSSION

Chloroquine and HCQ are well-known drugs and have been used for decades as antiparasitic and anti-inflammatory drugs to treat malaria and rheumatological disorders. Chloroquine was shown to be effective against SARS-CoV in invitro studies. This may be because of disruption of viral replication, changing immune system activity in addition to its inflammatory effect.^17^

The two drugs have been tried earlier for the treatment of SARS infection and showed promising efficacy. With the emergence of SARS-CoV-2 pandemic, they have been suggested as potential treatment for the new coronavirus 2019 based on the previous evidence from different coronavirus strains.^18^

Although cardiac toxicity is a known adverse event requiring monitoring during treatment, HCQ showed promise in treating SARS-CoV-2–infected patients with multiple comorbidities including coronary artery disease. A large trial from India showed that HCQ can decrease time to recovery both in symptomatic and in asymptomatic patients with no effect on mortality.^19^

At the beginning of the pandemic in Europe, a small series of COVID-19 patients treated in France with HCQ showed improved decline in SARS-CoV-2 viral load compared with controls, which was augmented by the addition of azithromycin.^7^ However, this study had serious methodological flaws and could not be considered as a good evidence in the favor of HCQ use.^8–11^

Many other conflicting trials have been published in the past few months leading initially to emergency use authorization for HCQ use in the treatment of COVID-19 and later on withdrawal of this authorization by the FDA. Initial observational trials of HCQ use in hospitalized patients showed that there were no increased risks of mortality or intubation in groups receiving HCQ or the control group who received only standard of care although patients who received HCQ were more critically ill.^20^ However, many published trials had some methodological flaws and missed important patient outcomes urging the need for properly designed, adequately powered trials to support clinical decisions of HCQ use in treating COVID-19 patients.^21^

Administration of HCQ did not result in a significantly higher probability of conversion from positive to negative PCR than standard care alone in patients admitted to hospital with nonresponsive mild-to-moderate COVID-19 in China. Adverse events were more frequent in HCQ recipients than in non-recipients.^22^

A meta-analysis included seven studies with a large number of patients showing that treatment with HCQ was associated with faster improvement of fever, cough, and less radiological progression of lung lesions. However, there was no difference in the virological cure, clinical improvement, or mortality.^23^

Many subsequent trials did not show benefit for HCQ use in COVID-19, with some of them suggesting more adverse events associated with its use.^22–24^ A recent clinical trial by Skipper et al.^12^ studied the change in symptom severity over 14 days in nonhospitalized patients between HCQ and control groups and did not find any significant difference (*P* = 0.12). Another trial by Cavalcanti et al.^13^ compared three groups; standard care group, standard care plus HCQ, and standard care plus HCQ and azithromycin. The clinical status at 15 days assessed by a seven-level ordinal scale did not show any significant difference among the three groups. Moreover, elevated liver enzymes and prolonged QT intervals were more frequent among patients who used HCQ.

In our study, adding HCQ to standard care did not add an extra benefit for the patients. Hydroxychloroquine arm was similar in all outcomes. Moreover, HCQ was not effective as postexposure prophylaxis against COVID-19 when administered within 4 days after exposure.^25–29^

Limitations of the study include small sample size which was not adequately powered for survival endpoint. The number of the included patients was limited because in Egypt, tertiary care hospitals were assigned lately to deal with COVID-19 patients and had many regulations by the Egyptian MOH. The study lacks long-term follow-up which could be addressed in a prospective trial. The utility of HCQ should be evaluated in larger multicenter trials either alone or in combination with other drugs/lines of treatment. The role of HCQ as a prophylaxis against SARS-CoV-2 infection should be among the future trials also.

In conclusion, our trial adds extra evidence from Egypt that HCQ may not be beneficial as a treatment for COVID-19.
